# Effects of Acupuncture on Neuropathic Pain Induced by Spinal Cord Injury: A Systematic Review and Meta-Analysis

**DOI:** 10.1155/2022/6297484

**Published:** 2022-08-19

**Authors:** Kelin He, Rong Hu, Yi Huang, Bei Qiu, Qinqin Chen, Ruijie Ma

**Affiliations:** ^1^Department of Acupuncture and Moxibustion, The Third Affiliated Hospital of Zhejiang Chinese Medical University (Zhongshan Hospital of Zhejiang Province), Hangzhou, Zhejiang, China; ^2^Key Laboratory of Acupuncture and Neurology of Zhejiang Province, The Third School of Clinical Medicine (School of Rehabilitation Medicine), Zhejiang Chinese Medical University, Hangzhou, Zhejiang, China

## Abstract

**Introduction:**

Neuropathic pain is a commonly seen symptom and one of the most intractable comorbidities following spinal cord injury (SCI). Acupuncture has been widely used for neuropathic pain after SCI in clinical settings. There is no systematic review or meta‐analysis evaluating the efficacy of acupuncture in the treatment of SCI-induced neuropathic pain. Thus, this study aimed to conduct a systematic review and meta-analysis to assess the efficacy of acupuncture on SCI-induced neuropathic pain.

**Methods:**

Seven databases were comprehensively searched, including PubMed, the Cochrane Library, the Web of Science, the China National Knowledge Infrastructure (CNKI), the Chinese Biomedical Literature Service System (SinoMed), the Wanfang Database, and the Chinese Scientific Journals Database (VIP) from their inception to 30 September 2021. Two independent reviewers evaluated the eligibility of the data retrieved based on the pre-established eligibility criteria and assessed the methodological quality of the included studies using the Cochrane Risk of Bias Tool. The outcome indexes in this study included the visual analogue scale, the numeric rating scale, the present pain intensity, and the pain region index. Sensitivity and subgroup analyses were also performed to specifically evaluate the intervention effects. In addition, publication bias was analyzed.

**Results:**

Six randomized controlled trials (145 participants in the experimental groups and 141 participants in the control groups) were identified that evaluated the application of acupuncture for neuropathic pain after SCI and were included in this study. The results of our study revealed that acupuncture had a positive effect on the pain severity (standardized mean difference (SMD): −1.40, 95% confidence interval (CI): −2.23; −0.57), the present pain intensity (MD = −0.61, 95% CIs = −0.98; −0.23), and the pain region index (MD = −3.04, 95% CI = −3.98; −2.11). In addition, sensitivity analyses showed that these results were robust and stable. Subgroup analyses indicated that electroacupuncture (EA) had better effects on SCI-induced neuropathic pain. However, a publication bias was observed.

**Conclusion:**

Available evidence appears to suggest that acupuncture may have a role in SCI-induced neuropathic pain management, but this remains to be determined.

## 1. Introduction

Neuropathic pain is a commonly seen symptom and one of the most intractable comorbidities of spinal cord injury (SCI), affecting patient satisfaction and quality of life. Each year, an estimated 250,000 to 500,000 SCI cases are diagnosed around the world, more than 90% of them are due to trauma injury [1], and about 30–50% of patients with SCI will experience chronic neuropathic pain [2, 3]. However, neuropathic pain remains a substantial clinical and economic burden and therapeutic challenge. It has been estimated that, on average, $47,518 is spent for every SCI patient with neuropathic pain in the United States of America [4]. Currently, available treatments for SCI-induced neuropathic pain are limited in clinical practice. Methods commonly applied to relieve neuropathic pain involve western approaches that primarily include drugs and mini-invasive stimulation. The agents frequently used in treating neuropathic pain include pregabalin and gabapentin [5]. However, these drugs are often ineffective, or just effective for a small number of participants, and even have side effects [6]. Mini-invasive stimulation, such as spinal cord stimulation, has been widely used to manage neuropathic pain [7, 8]. However, there is no significant evidence supporting this approach for participants with SCI experiencing neuropathic pain [9]. Therefore, there is a strong demand to develop novel and effective therapies for neuropathic pain due to SCI.

Acupuncture, as an integral part of traditional medicines around the world for the treatment of acute and chronic pain, has recently attracted widespread attention. It is increasingly being applied in scientific and clinical research [10–13]. The mechanism of acupuncture analgesia, including opioids, *γ*-aminobutyric acid (GABA), signaling pathways, and the immune system, is being increasingly elucidated in recent years [14]. In addition, acupuncture-induced analgesia may act on different levels of the nervous system, including the spinal cord and the brain [15–17]. In addition, there is an international consensus on acupuncture treatment for analgesia in clinical practice [18]. Recently years, acupuncture has been widely used for patients with SCI, not only for neurological dysfunction but also for neuropathic pain [19]. However, the clinical efficacy of acupuncture in SCI-induced neuropathic pain remains uncertain. To date, many clinical studies on the treatment of neuropathic pain with acupuncture have been reported [20–22]. However, no relevant systematic reviews or meta-analyses have been performed to address the efficacy of acupuncture in SCI-induced neuropathic pain. Therefore, we conducted a systematic review and meta-analysis to evaluate the effectiveness of acupuncture in treating neuropathic pain after SCI. This study may help to provide guidelines for future prospective clinical application of acupuncture therapy for neuropathic pain subsequent to SCI.

## 2. Methods

### 2.1. Design

This present study followed the Preferred Reporting Items for Systematic Reviews and Meta-Analyses (PRISMA) guidelines [23], and the study protocol was registered at https://inplasy.com/ (registration number: INPLASY2021100107).

### 2.2. Search Strategy

We systematically searched the following seven electronic databases from inception to 30 September 2021: PubMed, the Cochrane Library, the Web of Science, the China National Knowledge Infrastructure (CNKI), the Chinese Biomedical Literature Service System (SinoMed), the Wan-fang Database, and the Chinese Scientific Journals Database (VIP), to identify all randomized control trials (RCTs) on acupuncture in treating SCI-induced neuropathic pain. The following terms were searched as subject words, keywords, free-text terms, and MeSH terms: spinal cord injuries, spinal cord injury, neuropathic pain, neuralgia, acupuncture, acupuncture therapy, electroacupuncture, warming needle moxibustion, fire needling, fire needle, and fire acupuncture. Apart from the above, there were no restrictions on language, region, or country.

### 2.3. Eligibility Criteria

This study included all available RCTs investigating acupuncture for the treatment of neuropathic pain after SCI. All other types of literature such as system reviews, letters, case reports, editorials, animal studies, commentary, and non-RCTs were excluded.

### 2.4. Participants

This study only included studies that involved adult participants (>18 years of age) diagnosed with SCI-induced neuropathic pain. The following studies were excluded: SCI caused by tumor, infection, or autoimmune disorders.

### 2.5. Interventions

The intervention in the experimental group included acupuncture alone or in combination with conventional therapy, and the control group included conventional treatment and/or sham acupuncture.

### 2.6. Outcomes

The primary outcome indicator of this study was pain severity, and the secondary outcome indicators included the present pain intensity and pain region index.

### 2.7. Literature Selection and Data Extraction

One reviewer (Rong Hu) performed the literature search according to the pre-established search strategy and downloaded the related citations. All literature studies were imported into Endnote X9 software, and duplicate studies were removed using electronic/manual checking. Subsequently, two independent reviewers (Rong Hu and Bei Qiu) screened and identified the titles and abstracts of the remaining literature and then independently retrieved the studies that fulfilled the inclusion criteria. Inconsistent results between reviewers were resolved by discussion or by involving the corresponding author. After the initial screening, two reviewers independently extracted the following information from the identified studies: general information (authors, publication year, and country), demographic data (sample size, intervention, age, sex, onset of SCI, ASIA grade, and spinal segment), acupuncture protocol (acupoints, acupuncture modality, retention time, and treatment duration), and outcome measures.

### 2.8. Data Analysis

#### 2.8.1. Assessment of Risk of Bias in the Included Studies

Two independent reviewers (Qinqin Chen and Yi Huang) evaluated the bias risk of each study by using the Cochrane risk of bias assessment tool [24]. This assessment tool mainly included seven domains: random sequence generation, allocation concealment, blinding of participants and personnel, blinding of outcome assessment, incomplete outcome data, selective reporting, and other sources of bias. Each domain of the individual study was classified as high, low, or unclear risk. Any discordance between the two reviewers was resolved by discussion with the corresponding author.

#### 2.8.2. Statistical Analysis

All data analyses of this study were performed using the R software (version 3.6.3; package meta). Continuous variables were calculated as mean differences (MD) and 95% confidence intervals (CI). If MD measurements varied between studies, a standardized MD (SMD) was calculated for meta-analyses. The *I*^2^ statistic was used to evaluate the heterogeneity of the studies (with *I*^2^ statistic > 50% indicating statistically significant heterogeneity). In addition, sensitivity analyses and subgroup analyses were carried out to detect the heterogeneity.

## 3. Results

### 3.1. Literature Selection

In total, 411 published references were initially identified (92 references from the CNKI, 109 references from the Wan-fang database, 21 references from the VIP, 101 references from the SinoMed, 19 references from PubMed, 21 references from the Cochrane Library, and 48 references from the Web of Science) and were imported into Endnote X9. After eliminating duplicates, 287 articles were retained. We further excluded reviews, case reports, animal experiments, and other irrelevant studies, and 22 studies remained. Moreover, mixed interventions, nonrandomized methods, missing data, and outcome indicators that did not include the primary or secondary outcomes were excluded. Finally, six RCTs were considered after reading the full-text articles. The detailed flowchart of the literature screening process is shown in Figure 1.

### 3.2. Characteristics of Included Studies

A total of six studies were included, which comprised 286 participants with neuropathic pain after SCI (141 participants in the control group and 145 participants in the experimental group). The interventions in the control group included conventional therapy only, and the interventions in the experimental groups included conventional therapy plus acupuncture. Of these, four studies did not report the ASIA grade of SCI. For the outcome measure, five trials involved the visual analogue scale, one trial involved the numeric rating scale, four trials involved the present pain intensity, and three trials involved the pain region index. The detailed characteristics of the included studies are shown in Table 1.

### 3.3. Risk of Bias Assessment

Figure 2 presents a summary of the bias risk of the included studies. Four trials reported random sequence generation and were assessed as having a low risk of bias [25, 26, 29, 30], two trials only mentioned “random” but without the description of the specific method used and were evaluated as unclear risk of bias [27, 28]. Nonetheless, all trials were not clear about the bias risk of the other six domains.

### 3.4. Meta-Analysis Results

#### 3.4.1. Meta-Analysis Results of Pain Severity by Visual Inspection

All trials involved pain severity. After carefully reading the full text of the corresponding studies, five trials used the visual analogue scale [25–29], and one trial used the numeric rating scale [30]. Hence, SMD was calculated for the meta-analysis. The result of the *I*^2^ statistic >50% and a random-effects model were used to perform the meta-analysis. Results showed that the acupuncture compared with no acupuncture intervention was significantly different (SMD = −1.40, 95% CIs = −2.23; −0.57), as shown in Figure 3(a). Subgroup analysis results showed that electroacupuncture (EA) had a larger positive effect size (SMD = −1.64, 95% CIs = −3.04; −0.23) than no EA treatment (SMD = −0.61, 95% CIs = −1.32; −0.09) on SCI-induced neuropathic pain (Figure 3(b)). In addition, the sensitivity analysis revealed that the result of this meta-analysis was robust.

#### 3.4.2. Results of the Meta-Analysis of the Present Pain Intensity

A total of four trials involved the present pain intensity [26–29]. The results of the *I*^2^ statistic >50% and the random-effects model were used to perform a meta-analysis. The meta-analysis results revealed a significant difference between acupuncture and no acupuncture effects (MD = −0.61, 95% CIs = −0.98; −0.23), as shown in Figure 4(a). The results of the subgroup analysis showed that Jiaji EA had a larger positive effect size (MD = −0.65, 95% CIs = −1.12; −0.19) than EA (MD = −0.80, 95%CIs = −1.38; −0.22) (Figures 4(b) and 4(c)). Furthermore, the sensitivity analysis revealed that the meta-analysis result was stable.

#### 3.4.3. Results of the Meta-Analysis of the Pain Region Index

A total of three RCTs used the pain region index [26–28]. The results of the *I*^2^ statistic = 31%; thus, a fixed-effects model was used to perform meta-analysis. The results of this meta-analysis showed that acupuncture compared with no acupuncture showed a significant outcome difference (MD = −3.04, 95% CIs = −3.98; −2.11) (Figure 5). Furthermore, the sensitivity analysis showed that the results of this meta-analysis were credible.

### 3.5. Publication Bias

Publication bias is a potential concern in meta-analyses when interpreting the meta-analysis results. In this study, the funnel plot and the trim-and-fill method were used to assess publication bias. A publication bias was indicated by an asymmetry funnel around the pooled effect size. Noteworthily, the selected studies did not lie symmetrically around the pooled effect size, and the trim-and-fill method also revealed evidence of publication bias (*p* < 0.05) (Figure 6).

## 4. Discussion

This could be the first meta-analysis to exclusively evaluate the effect of acupuncture on SCI-induced neuropathic pain. Six studies were included in our analysis, and the results indicated that acupuncture has a positive effect on SCI-induced neuropathic pain. When pooling these studies, a positive pooled effect size emerged (SMD = −1.40, 95% CI = −2.23, −0.57; *p* < 0.01). Of note, our findings revealed that EA may have better therapeutic efficacy on SCI-induced neuropathic pain. Therefore, our results may provide an important reference value for clinical investigation and provide essential information to decision-makers.

SCI-induced neuropathic pain has always been an intractable medical concern. Many studies have investigated whether acupuncture could be used as a therapeutic approach to SCI and its complications, and the results showed that acupuncture had a positive effect [31–33]. To date, the number of RCTs that investigated acupuncture as a therapeutic approach for SCI-induced neuropathic pain is very small. Therefore, it is not sufficient to offer credible estimates of the treatment effects. A systematic review is extremely helpful for combining results from these studies and to summarize the best research evidence available on a specific theme. However, to date, no literature review has been designed to specifically assess the efficacy of acupuncture on SCI-induced neuropathic pain. Our study could be the first meta-analysis to systematically assess the value of acupuncture in patients with neuropathic pain. The pooled effect size of −1.40 achieved statistical significance and was much higher than other previous meta-analyses of chronic neuropathic pain in adults [34]. However, there have been no relevant studies to date that involved the comparison of acupuncture and drugs, acupuncture, and mini-invasive stimulation. Consequently, significant differences between acupuncture and drugs and mini-invasive stimulation could not be determined. In addition, this study also underlines several potential elements that emerged from study outcomes and within and between-studies variances.

An important element to consider is the type of acupuncture treatment: EA versus no EA. This is the first study to compare these two treatments in an objective quantitative manner in an attempt to reach a definitive conclusion: what type of acupuncture treatment should be used? The results indicated that EA had larger pooled effect sizes on SCI-induced neuropathic pain. In many reviews, acupuncture was an effective treatment for alleviating chronic musculoskeletal, neck pain, headache, and osteoarthritis pain [35, 36]. Moreover, EA was the most common intervention in the treatment of chronic pain, which involved the application of an external electrical stimulus to acupuncture needles for acupoint stimulation [10, 36]. Basic research studies revealed that EA produced analgesic effects by activating or inhibiting a wide range of bioactive chemicals through peripheral and central mechanisms [10]. These include mobilization of human endogenous repair, inhibitory mechanisms (antioxidation, suppression of inflammatory cytokines, activation of the GABA inhibitory system, and descending inhibitory related brain areas) [37–39], and at the same time, inhibition of excessive activation of pathological pathways (excitatory ion channels, proinflammatory cytokines, glial cell activation, excitatory signal pathway, and activation of pain-related brain regions) [40–44]. Clinically, previous studies had shown that acupuncture could improve neurological recovery in patients with SCI [32], and EA was the main mode of treatment for patients with SCI. Animal studies also showed that EA could improve nerve regeneration and functional recovery in the rat model of SCI [45]. Currently, there are few reports on animal studies of EA on SCI-induced neuropathic pain in animal models, and the mechanism of EA has not yet been very clear. One study showed that EA was capable of markedly inhibiting mTOR signaling and blocking SCI-induced neuropathic pain in rats [46]. It should also be noted that Jiaji EA is frequently used among all EA methods. The Jiaji acupoint is located on both sides of the spine, and many studies choose Jiaji acupoint as the treatment of spinal injury [47, 48].

In addition, many other elements are quite evident in the studies that we analyzed. First, in the funnel plot, there was a significant degree of asymmetry, suggesting that there was a potential publication bias where “negative” studies were less likely to be reported. Prioritized published articles with differences between groups might be due to the rejection by journal editors of negative studies in this research field and seriously limits the effectiveness of acupuncture treatment. Second, most studies did not mention the ASIA grade of SCI, and only two studies reported the ASIA grade [27, 30]. According to a previous study, the ASIA grade on admission affected the subsequent recovery in both univariate and multivariate analyses [49]. Therefore, we could not explore the homogeneity of the ASIA grade included in the conditions. Third, the study by Irene et al. [30] reported a very long course of SCI; therefore, we could not establish whether there was a similar baseline for both groups. Fourth, there were many differences in the injured spinal segments between the affected individuals, and thus, this made it more complicated and difficult to interpret the effects of acupuncture on SCI-induced neuropathic pain. Furthermore, the randomization method is an important issue, as only four of our included studies mentioned specific randomization procedures, while the remaining two studies only mentioned that “participants were randomly assigned to two equal groups” with no further details provided. Thus, we believed that some of these studies were not real RCTs. A second caveat is that possible selection bias may originate in the vague inclusion/exclusion criteria and the selection of control groups in their study. No trial used sham acupuncture, and participants, clinicians, and outcome assessors in these studies were not blinded, all of which could have introduced information bias. Moreover, participants in clinical trials might have been enrolled because of expectations on pain improvement with acupuncture treatment. In addition, no trial provided information on withdrawals or dropouts or used intention-to-treat analysis. Furthermore, since only one study reported results up to the washout period, the long-term efficacy of acupuncture treatment could not be evaluated.

This study has several limitations that should be considered. First, the sample size of the studies included in this view was relatively small. As a result of the high clinical heterogeneity of SCI-induced neuropathic pain, clinical trials with large samples are particularly important. Therefore, meta-regression may be needed to adjust these variables; however, the small sample size of those studies makes it unachievable. Second, although a comprehensive literature search was conducted using multiple online databases, it remains possible that some eligible studies may still have been missed in our search. Third, the absence of ASIA grades in most studies limited our ability to analyze the effects of acupuncture on SCI-induced neuropathic pain in different ASIA grades. In addition, due to the lack of placebo acupuncture in the control group, we were unable to analyze the difference in the curative effects between acupuncture and sham acupuncture.

## 5. Conclusions

In conclusion, acupuncture may have a positive role in the management of SCI-induced neuropathic pain. However, small sample sizes, variable methodological quality, and heterogeneity in study design weaken these inferences. Therefore, more high-quality studies are needed in the future.

## Figures and Tables

**Figure 1:** Flow diagram depicting the selection process of eligible studies (CNKI, China National Knowledge Infrastructure; VIP, Chinese Scientific Journals database; SinoMed, Chinese Biomedical Literature Service System; *n* number of publications).

**Figure 2:** Risk of bias of all included studies.

**Figure 3:** Forest plots of the pain severity by visual inspection. (a) Overall analysis of the six included trials; (b) subgroup analysis based on the acupuncture mode (EA vs. no EA).

**Figure 4:** Forest plots of the present pain intensity. (a) Overall analysis of the four included trials; (b) subgroup analysis of EA; (c) subgroup analysis of Jiaji EA.

**Figure 5:** Forest plots of the pain region index.

**Figure 6:** Meta-analysis results of publication bias.

**Table 1:** Characteristics of the included studies.

Study	Publicationyear	Country	Sample		Intervention		Age (years)		Sex (M/F)		Onset of SCI		ASIA grade	Injured spinal segments	Acupunctureprotocol	Outcome measure
			C	E	C	E	C	E	C	E	C	E				
Zheng et al. [25]	2021	China	35	35	Rehabilitative + drug	Rehabilitative + drug + acupuncture	36.35 ± 10.82	38.48 ± 11.40	18/17	20/15	(5.08 ± 0.84) (m)	(4.64 ± 0.68) (m)	Not mentioned	Cervical, thoracic, and lumbar region	Electroacupuncture (2 Hz) at “Jiaji” (EX-B2) + scalp acupuncture at the motor, sensory, spiritual, and emotional areas of Jiao's; the treatment duration was 30 minutes, once a day for 28 consecutive days	VAS
Cheng [26]	2018	China	27	27	Drug	Drug + acupuncture	47.98 ± 5.27	48. 16 ± 5.12	18/9	17/10	(4.91 ± 1.05) (m)	(5.11 ± 0.87) (m)	Not mentioned	Cervical, thoracic, and lumbar region	Electroacupuncture (sparse and dense waves) at “Jiaji” (EX-B2); the treatment duration was 30 minutes, once a day for 25 consecutive days	VAS, PRI, PPI
Chen et al. [27]	2014	China	18	18	Drug	Acupuncture	18–62		20/16		With a minimum of 2 months and a maximum of 50 years		ABCD	Cervical, thoracic, and lumbar region	Electroacupuncture (sparse and dense waves) at “Governor Vessel” acupoints; the treatment duration was 30 minutes, once a day for 30 consecutive days	VAS, PRI, PPI
Chen et al. [28]	2015	China	23	23	Rehabilitative + drug	Rehabilitative + drug + acupuncture	38.2 ± 9.6		20/26		(2.5 ± 0.8) (m)		Not Mentioned	Not mentioned	Acupuncture at Baihui (GV 20), He-Gu (LI4), and Ashi points, 6 times a week for 4 weeks	VAS, PRI, PPI
Fang et al. [29]	2016	China	30	30	Drug + massage	Drug + massage + acupuncture	38.2 ± 6.1		44/16		(3.8 ± 0.4) (m)		Not mentioned	Not mentioned	Electroacupuncture at “Jiaji” (EX-B2); the treatment duration was 30 minutes, once a day for 20–30 days based on clinical need	VAS, PPI
Irene et al. [30]	2017	USA	8	12	Rehabilitative + drug	Rehabilitative + drug + acupuncture	46.1	41.1	6/2	10/2	13 years	7.6 years	ABCD	Not mentioned	Auricular acupuncture at the anterior cingulate, thalamus, omega-2, Shen Men, point zero; the treatment duration was 3-7 days, once a week for 8 weeks	NRS

m, months; C, control group; E, experimental group; VAS, visual analogue scale; NRS, numeric rating scale; PPI, present pain intensity; PRI, pain region index.

## Data Availability

All data relevant to the study are included in the article.
